# Research on the Implementation of Public Physical Education under the Network Environment

**DOI:** 10.1155/2022/6391614

**Published:** 2022-03-27

**Authors:** Chao Hong, Jie Ren

**Affiliations:** ^1^School of Department of PE, Dankook University, Yongin-si, Republic of Korea; ^2^Sports Department, Guilin Medical University, Guilin, China

## Abstract

In order to improve the physical quality of contemporary students, the public physical education teaching of big data technology is introduced to enrich the interest of physical education classroom and improve the enthusiasm of students through targeted teaching means. In this paper, through the big data of students' physical performance and students' physical quality, an expert system for physical education curriculum recommendation is established to teach students according to their aptitude and increase the intelligent management of the classroom. The SPSS simulation experiment is carried out according to the big data of students' physical performance and physical quality. Finally, it is concluded that the system can improve students' interest in physical exercise, increase the vividness of the classroom, and improve students' physical quality.

## 1. Introduction

At present, due to the development of society and economy, teachers and parents pay attention to students' achievements, which leads to the great academic pressure of current students and the overload of teaching and homework inside and outside class. Therefore, today's students have more and more close vision and younger age due to the extension of desk study time. As one of the compulsory courses for students, the purpose of physical education is to combine work and rest and maintain good physical and mental health development while learning. The state has repeatedly emphasized on the reform of student education that the all-round development of comprehensive quality is to separate students from the sea of questions, change from passive learning to active learning in combination with their own interests, and improve students' quality. In the era of Internet plus, deep learning and machine learning are introduced into the educational reform, and students are designed to take physical education courses.

The emergence of information technology provides modern tools for teaching. This paper points out that physical education combined with modern big data technology has become a scientific activity. In view of the problems encountered in the practice of physical education, this paper analyzes the auxiliary teaching of big data in middle school physical education and puts forward suggestions for promoting the application of big data in physical education in the future [1].) Colleges and universities have more teaching resources than middle schools. In the process of teaching, they also pay more attention to the application of high technology, and information technology promotes the development of physical education to fine teaching. This paper constructs the information system of physical education in colleges and universities through information as the carrier and effectively improves the efficiency of physical education through this system [2]. The above literature also highlights that teaching with the help of scientific and technological means is the characteristic of the current education reform. The use of scientific and technological means to teach students not only improves the quality of teaching, but also stimulates students' initiative in learning. According to the scientific planning of sports, the limited time in the classroom allows students to not only get the actual effect of exercise, but also enjoy the fun of sports.

There are still many deficiencies in the current physical education in colleges and universities. This paper studies these theoretical education to further optimize the theory of physical education, so as to promote the development of physical education in colleges and universities in the future [3].

Traditional sports are relatively rigid, lack of active guidance to students, and cannot stimulate students' interest, resulting in low classroom efficiency. In view of this characteristic, this paper introduces big data information to mine students' interests and laws, reforms according to the teaching content, and uses big data to carry out real-time teaching of physical education.

### 1.1. New Technology of the Internet Plus Background in Public Physical Education Teaching

#### 1.1.1. Big Data of Students' Sports Scores

By constructing the big data platform of students' sports performance, the test results of students' sports performance are input into the platform. The test result is that the school tests the students through sports and gives the test results to the students with the scoring system. The average value of students' various items reflects students' comprehensive sports performance, and the advantages of students' different items also reflect the preference of physical fitness and interest. According to this characteristic, students can develop their interests and expertise, so as to guide students' enthusiasm for physical education and improve the effectiveness of the classroom [4].

#### 1.1.2. Big Data of Students' Physical Quality

The big data of students' physical quality constructed can carry out targeted physical education according to the characteristics of students' physical quality. Because the physical quality of students is affected by family environment and genetic factors, they show different functions such as strength, speed, sensitivity, and flexibility. Their physical quality reflects their endurance and flexibility in learning and labor. According to these characteristics of students, targeted teaching can give better play to students' strengths and the purpose of exercise [5].

The function of physical education course recommendation expert system is to generate course recommendation information by using neural network method according to the specific data of students in the above two big data, so as to provide these students with the most suitable physical education elective courses. The specific algorithm used in the physical education course recommendation expert system is fuzzy neural network. The specific steps of the algorithm are to execute polynomial fuzzy neural network on two big data, respectively, build logarithmic multi column neural network for each elective course, and post binary neural network for each column. When the output is 1, the course is recommended, and when the output is 0, the course is not recommended.

## 2. Materials and Methods of Teaching Experiment

### 2.1. Selection and Grouping Methods of Students

Students in junior high school, senior high school, and university are selected as the research objects. Different physical education activities are opened according to different age groups, and the age span is relatively long. Between the ages of 12 and 27, the average age of men is 19.23 ± 2.5, the average age of women is 18.92 ± 1.9, and the ratio of men to women is about 1.12:1. Students participating in physical education are required to be healthy, have no obvious physical disability, and can complete classroom teaching independently. Exclude patients with cardiopulmonary insufficiency, indirect mental disorders, chronic diseases, and other diseases that are not suitable for vigorous action according to the doctor's advice.

Among them, 587 junior middle school students, 313 boys and 274 women; 512 high school students, 273 boys and 239 women; and 627 college students were selected, 334 boys and 293 women.

### 2.2. PE Elective Program and Course Selection Compliance

Football, basketball, volleyball, table tennis, badminton, Changquan routine, and Taijiquan routine are commonly used in physical education. Combined with the current situation and interests of teenagers, these items are selected for sports application, so as to achieve the purpose of creating group cooperation among students while exercising and developing the cohesion between students [6] .

When students choose the recommended courses given by the “physical education curriculum recommendation expert system,” they will be included in the compliance group, otherwise they will be included in the noncompliance group [7];

### 2.3. Teaching Application of PE Course Recommendation Expert System

Through the big data of students' physical performance and the big data of students' physical fitness, the polynomial fuzzy neural network is implemented for the two big data, respectively, and the logarithmic multicolumn neural network is constructed for each elective course to obtain the physical education course suitable for each student, which increases the vividness and interest of the classroom, thus affecting students' active participation in physical exercise, strengthen students' physical quality, and improve students' physical performance [8].

### 2.4. Observation Contents and Methods

This paper analyzes the impact of elective courses based on big data on physical performance and students' physical quality through the passing rate of football, basketball, volleyball, table tennis, badminton, Changquan routine, and Taijiquan routine examinations of boys and girls [9]. At the same time, observe the test compliance rate of students who follow the courses pushed by big data and those who do not, the change of students' enthusiasm for extracurricular sports activities, and the change of physical quality. Recommend courses through students' performance big data and physical quality big data to increase the interaction between teachers and students in the classroom, so as to improve physical quality. Effective detection of students' academic performance is the most commonly used method to assess learning. Through normal physical education test and physical fitness test, the assessment results are used to distinguish the impact of elective courses based on big data on students' physical quality [10].

The observation method used in this paper is to statistically analyze the final physical examination scores of students in compliance group and noncompliance group and analyze the data with bivariate *t* and *P* [11].

### 2.5. Statistical Method

The neural network module adopts polynomial depth iterative regression node function, and its basis function is written in formula (1)

(1) $$\begin{array}{c} y=\overset{n}{\underset{i=1}{\sum }}\overset{5}{\underset{j=0}{\sum }}A_{j}x_{i}^{j}, \end{array}$$

where *x*_*i*_^*j*^ is the *j*th power of the input value of the *i*th node in the upper neural network; *A*_*j*_ is the coefficient to be regressed of the *j*th order polynomial; and *n* is the number of nodes of the upper neural network.

The node basis function of the binary neural network is shown in formula (2)

(2) $$\begin{array}{c} y=\overset{n}{\underset{i=1}{\sum }}\frac{1}{A+B\cdot e^{x_{i}}}, \end{array}$$

where *e* is the natural constant and the approximate value *E* = 2.718281828 is taken; other mathematical symbols have the same meaning as formula (1) above;

*t-Calibration*. The counting data is expressed in (%), chi-square test and analysis of variance are used according to the nature of the data, and spss24 used 0 statistical analysis software. Only the calculation algorithm of *T* value (value value) is explained here, such as formula (3)

(3) $$\begin{array}{c} t_{\text{Value}}=\frac{\bar{x}-\mu }{S/\sqrt{n-1}}, \end{array}$$

where $\bar{x}$ is the arithmetic mean of the sample series of physical education model; *μ* is the average value of the sample series of previous physical education models; *n* is the number of nodes in this series of physical education mode; *m* is the number of nodes in the sample sequence of previous physical education models; and *S* is the standard deviation rate of physical education sample sequence.

The algorithm for calculating the average value in formula (3) is shown in formula (4)

(4) $$\begin{array}{c} \bar{x}=\frac{1}{n}\overset{n}{\underset{i=1}{\sum }}x_{i}, \end{array}$$

where *i*  is traversal pointer; *m* is the number of nodes in the sample sequence of previous physical education models; and *x*_*i*_ is the *i*th input value in the sequence; the meaning of mathematical symbols is the same as before.

The algorithm of standard deviation rate in formula (3) is shown in formula (5)

(5) $$\begin{array}{c} S=\frac{1}{n-1}\sqrt{\overset{n}{\underset{i=1}{\sum }}{\left(x_{i}-\bar{x}\right)}^{2}}. \end{array}$$

## 3. Observation Results of Teaching Experiment

### 3.1. Influence of Different Elective Courses on Students' Physical Education Performance

Track and record all the students participating in the experiment, observe the compliance of the compliance group and noncompliance group participating in different physical education elective courses, and record and analyze the data in Table 1.

In Table 1, the difference between different groups was statistically significant (*P* < 0.05). It can be seen from the data in the above table that there is no significant difference between boys and girls in the examination compliance rate of different sports, but for the same project, the compliance rate of students in the compliance group is much higher than that in the noncompliance group, which shows that the recommended courses given by the “physical education course recommendation expert system” are targeted, it is scientific, suitable for different individual physique, and can be adopted to help students choose sports suitable for themselves. According to the data in Table 1, Figures 1 and 2 are separately compared and analyzed.

In Figure 1, all boys who follow the sports items recommended by the “physical education course recommendation expert system” have a compliance rate of more than 80% at the end of the term, while most of the students who do not follow the system's recommendation have a compliance rate of less than 60% at the end of the term, which shows that the physical education subjects recommended by the system are beneficial to the improvement of boys' physical education examination results.

Figure 2 shows the data of the standard rate of physical examination scores of all girls participating in the experiment. Like the law of boys, the standard rate of physical examination scores of girls in the compliance group is much higher than that in the noncompliance group. This shows that no matter boys or girls, as long as they follow the physical education elective courses recommended by the system, they are easier to pass the physical education examination than those who do not follow.

### 3.2. Effects of Different Elective Courses on Students' Physical Quality

The physical fitness test scores of all students are counted and statistically analyzed to obtain the data in Table 2.

In Table 2, the comparison of the physical fitness test compliance rate data of students in different physical education subjects has statistical significance (*P* < 0.05). It can be seen from the data in the table that the physical fitness test achievement rate of both boys and girls is much higher than that of students who do not follow the physical education subjects recommended by the system. This shows that the physical education subjects recommended by the system can enhance students' physique, so the physical fitness test score will be high. According to the data in Table 2 above, as shown in Figures 3 and 4, the data can be analyzed from the perspective of gender.

In Figure 3, for the students who follow the physical education subjects recommended by the system, the compliance rate of their comprehensive physical fitness test is more than 95%; for students who do not comply with the recommendation of the system, their physical fitness test compliance rate is not satisfactory. Most of the compliance rate is about 75%, and the compliance rate of the compliance group is about 20% higher than that of the noncompliance group, which shows that the physical fitness of boys in the compliance group is far better than that of boys who do not comply with the system and indirectly shows that the use of the system can improve the physical fitness of boys.

In Figure 4, as in the case of boys, the compliance rate of girls' physical fitness test in the compliance group is also much higher than that in the noncompliance group, which shows that the system is suitable for both boys and girls. It can select appropriate physical education courses for them according to different individual differences, which is of great benefit to improve their physical quality.

## 4. Discussion on the Relationship between Course Selection Compliance and Students' Physical Education Performance

Carry out the implementation and use of the system for students of different ages, so as to analyze the sensitivity of students who accept the system to the age of use. Therefore, the statistical analysis of physical examination scores of students of different ages is shown in Figure 5.

As can be seen from Figure 5, the sports achievement standard rate of students of different ages is slightly different. With the increase of the years of accepting the system, the higher the sports achievement standard rate of students, which shows that the earlier the system is used, the better the improvement of students' sports achievement.

## 5. Discussion on the Relationship between Course Selection Compliance and Students' Physical Quality

Carry out the implementation and use of the system for students of different ages, so as to analyze the sensitivity of students who accept the system to the age of use. Therefore, carry out statistical analysis of physical examination scores for students of different ages and get the following Figure 6.

It can be seen from Figure 6 that the physical performance compliance rate of students of different ages is slightly different. With the increase of the service life of the system, the higher the physical performance compliance rate of students, which shows that the earlier the system is used, the more beneficial it is to improve students' physical performance and that the use of the system can improve students' physical quality.

## 6. Summary

Based on the Internet plus, the study introduced the big data technology and set up an expert system for PE curriculum recommendation aiming at the characteristics of the students themselves [12]. The aim is to recommend sports elective courses that meet their own characteristics and carry out sports activities, so that students can take part in sports activities actively and guide students to take the initiative to exercise with interest. And through the examination results to evaluate the impact of the system on students' physical performance and students' physical quality, it not only promotes the healthy development and growth of students, but also changes from the artificial and complex teaching environment to the process of science and technology teaching, reasonably plans and arranges physical education courses, improves students' enthusiasm, and increases the interaction between teachers and students, so as to improve the effectiveness of physical education teaching. At present, the introduction of big data technology into the teaching of colleges and universities at all levels is still in the experimental stage, and there are still deficiencies that need to be improved in practice to jointly help the development of education in the motherland.

## Figures and Tables

**Figure 1:** Comparison of PE examination standard rate of boys in different groups.

**Figure 2:** Comparison of PE examination standard rate of girls in different groups.

**Figure 3:** Comparison of physical fitness test compliance rate of boys in different groups.

**Figure 4:** Comparison of physical fitness test compliance rate of girls in different groups.

**Figure 5:** (Compliance/noncompliance) physical education achievement standard rate of students of different ages.

**Figure 6:** (Compliance/non-compliance) physical fitness test compliance rate of students of different ages.

**Table 1:** Comparison of PE examination standard rate of students in different groups.

Grouping	Schoolboy		Schoolgirl	
	Compliance	Noncompliance	Compliance	Noncompliance
Football	87.35	53.24	86.28	50.94
Basketball	89.58	49.61	88.47	48.37
Volleyball	88.92	55.68	89.31	53.72
Table tennis	90.87	60.38	88.82	56.91
Badminton	88.57	56.23	89.27	50.21
Long fist routine	81.62	48.94	82.37	47.15
Taijiquan routine	80.64	46.51	81.37	47.25

**Table 2:** Comparison of physical fitness test compliance rates of students in different groups.

Grouping	Schoolboy		Schoolgirl	
	Compliance	Noncompliance	Compliance	Noncompliance
Football	97.58	73.65	96.47	70.28
Basketball	97.16	74.58	96.38	71.31
Volleyball	98.47	78.36	97.41	74.13
Table tennis	96.58	74.17	95.19	76.28
Badminton	97.36	76.34	98.17	74.29
Long fist routine	98.59	79.21	97.79	73.48
Taijiquan routine	97.48	77.17	97.81	74.54

## Data Availability

The data underlying the results presented in the study are available within the manuscript.
